# Nursing of Vulvar Cancer Radical Operation Combined with Laparoscopic Inguinal Lymph Node Dissection

This article has been retracted.

**DOI:** 10.1155/2022/8091114

**Published:** 2022-09-05

**Authors:** Simei Huang, Feifei Qiu

**Affiliations:** Department of Anesthesiology, The Second Affiliated Hospital of Guangzhou University of Chinese Medicine, Guangzhou 510120, China

## Abstract

**Purpose:**

The application, development, and care of radical surgery combined with laparoscopic inguinal lymph node dissection for vulvar cancer.

**Methods:**

We searched the PubMed, Web of Science, the Cochrane Library, and EMBASE databases for published literature on the care of radical surgery combined with laparoscopic inguinal lymph node dissection for vulvar cancer up to June 2022. We used the following search terms and terms: “vulvar cancer,” “injury,” “radical vulvar cancer surgery,” “laparoscopic inguinal lymph node dissection,” and “care.”

**Results:**

Laparoscopic inguinal lymph node dissection has become a new surgical method for the treatment of vulvar cancer, and it effectively avoids all the problems associated with traditional surgery. In addition, radical vulvar cancer surgery and laparoscopic inguinal lymph node dissection combined with high-quality nursing interventions can promote patients' recovery and reduce the occurrence of complications, which has important clinical significance.

**Conclusion:**

This article reviews the application, development, and nursing care of radical vulvar cancer surgery combined with laparoscopic inguinal lymph node dissection.

## 1. Introduction

Vulvar cancer is a relatively rare malignant tumor of female genital organs, accounting for about 3%–5% of female genital tumors, and it occurs in people over 60 years old [1]. The pathogenesis of vulvar cancer is unclear [2]. Studies have shown that the occurrence of vulvar squamous carcinoma is associated with human papillomavirus (HP) infection, vulvar nonneoplastic epithelial lesions, such as vulvar sclerosing moss, and sexually transmitted diseases [3]. Lymph node metastasis is an important risk prognostic factor for vulvar cancer. Therefore, lymphadenectomy (IL) is an important part of the surgical procedure for vulvar cancer. Although this procedure can provide better tumor control, the traditional open inguinofemoral lymphadenectomy (OIL) has a large surgical area, bleeding, and is prone to surgical site infection and necrosis, and postoperative complications are quite high, mainly including skin infection, necrosis, and laceration in the inguinal area, lymphatic leakage, lymphatic cysts, and lymphoma of the lower extremities. Postoperative complications include skin infection, necrosis, laceration, lymphatic leakage, lymphatic cysts, and lymphedema of the lower extremities, which seriously affect the recovery and quality of life of patients, and even affect the subsequent treatment of patients and reduce their efficacy, with some literature reporting up to 50% or more [1, 2, 4].

Although a series of improvements in surgical approaches have led to a decrease in the incidence of postoperative complications, the results have not met expectations. With the increasing rise of minimally invasive concepts in cancer treatment, laparoscopic inguinal lymph node dissection has become a new surgical procedure applied in the treatment of vulvar cancer, which has been reported at home and abroad. Laparoscopic inguinal lymph node dissection has the advantages of less trauma, less bleeding, less interference with the physiological functions of tissues and organs, less postoperative pain, faster recovery, less surgical scar, and less impact on immune function. It can effectively avoid the most common problems of skin necrosis in the inguinal region and poor long-term healing of the incision, reduce complications, and significantly improve patients' quality of life [5–7].

It is clinically important to carry out a quality nursing approach from the actual situation of patients to give them comprehensive rehabilitation care and promote their recovery. Preoperative psychological care, adequate preoperative preparation, postoperative incision observation and care, functional exercise, and prevention of complications are especially important for patients' recovery. Therefore, quality nursing interventions for radical vulvar cancer combined with laparoscopic inguinal lymph node dissection can promote patients' recovery, shorten the operation time, reduce the occurrence of complications, and improve the cure rate of patients, which is of great clinical significance (Figure1). This article reviews the application, development, and nursing modalities of radical vulvar cancer surgery combined with laparoscopic inguinal lymph node dissection. One hundred and twenty-one articles were read, of which 45 were RCTs and 11 were recommendations. Only 13 RCTs and 8 recommendations remained (Figure 2).

## 2. Overview of Vulvar Cancer

Vulvar cancer is a rare malignant tumor of the female reproductive system, accounting for only 2% to 5% of all malignant tumors of the female reproductive system. The incidence of vulvar cancer increases with age and is common in older women over the age of 75, especially postmenopausal women.

Vulvar cancer can be divided into two categories: vulvar cancer associated with HPV infection and vulvar cancer unrelated to HPV infection, the latter being mostly in young women and possibly combined with vulvar intraepithelial neoplasia (VIN). One study showed that high-risk HPV-DNA types were detected in approximately 40.1% of vulvar cancer patients, 80.4% of VIN-2, VIN-3, and 77.5% of VIN-1 patients, with HPV types 16, 18, 23, and 31 being the most common. In contrast, HPV-negative vulvar cancers are associated with intraepithelial nonneoplastic degeneration of the vulva (NNED), a group of chronic diseases characterized by degeneration of the mucosal tissue of the vulvar skin and pigmentary changes of vulvar pruritus, mainly including sclerosing lichen sclerosis (LS) and squamous epithelial hyperplasia of the vulva (SH). Patients with LS have a 4% to 6% risk of developing vulvar cancer. In addition, sexually transmitted diseases, herpes simplex virus infection, smoking, alcohol abuse, obesity, hypertension, diabetes, early sexual intercourse, and low social status may be associated with the development of vulvar cancer but are not independent risk factors [8, 9].

The most common pathological type of vulvar cancer is squamous cell carcinoma, which accounts for about 80%–90% of cases, followed by malignant melanoma, adenocarcinoma, basal cell carcinoma, verrucous carcinoma, and sarcoma. According to the degree of histological differentiation, they can be classified as hypodifferentiated, intermediately differentiated, and highly differentiated. The earlier the stage, the higher the survival rate and the better the prognosis. Improving the early diagnosis rate of vulvar cancer is an important factor to improve its prognosis [10] (Table 1).

From Table 1, we can see that much evidence proves that the early diagnosis rate of vulvar cancer is an important factor in improving its prognosis, and the earlier the diagnosis, the earlier the treatment, the higher the survival rate, and the better the prognosis.

### 2.1. Treatment of Vulvar Cancer

The treatment of vulvar cancer is mainly surgical, and individualized surgical methods and radiotherapy plans are selected according to the disease, tumor stage, and physical condition [11, 12]. If it is an early-stage vulvar cancer, surgical treatment can be used, and the specific surgical method should be decided according to the stage. In the case of stage 1a vulvar cancer, local expanded vulvar excision can be used, and in the case of stage 1b vulvar cancer, the surgical approach should be decided according to the specific location of the cancer lesion. If it is a unilateral lesion, extensive local excision or modified extensive vulvectomy can be performed, and unilateral inguinal lymph node dissection is also required. If it is a midline vulvar cancer, local wide vulvectomy and bilateral inguinal lymph node dissection are required. In the case of locally advanced tumors, the extent of surgery should be evaluated on a case-by-case basis and may need to be combined with adjuvant therapy, such as radiotherapy, after surgery. In the case of advanced cancer with distant metastases, chemotherapy and targeted therapy may be required, depending on the patient's condition.

Radical vulvar cancer surgery is a surgical procedure to treat cancer of the vulva and inguinal lymph nodes and includes combined radical vulvar cancer surgery and radical vulvectomy. The Way radical vulvectomy, also known as the Way procedure, is a simultaneous extensive vulvectomy and bilateral inguinal resection with sequential pelvic-iliac fossa lymph node dissection if necessary. The Way procedure remains the classic standard procedure for the treatment of intermediate to advanced vulvar cancer. Inguinal lymph node dissection is a term published in urology in 2014. It is a procedure in which all lymph nodes and the surrounding fat pad in the inguinal region are removed. It is mainly used to treat inguinal lymph node metastases from malignant tumors, such as penile cancer [13, 14].

Radiotherapy is often used as a preoperative or postoperative adjuvant treatment for vulvar cancer or as part of a comprehensive treatment for advanced vulvar cancer or advanced lesions to reduce the trauma of ultraextensive surgery and improve the prognosis of patients with vulvar cancer [15, 16]. Radiation therapy is not usually the first choice for vulvar cancer treatment, but it is an important part of the comprehensive treatment of vulvar cancer and is usually used in patients with lymph node metastases or in patients who are inoperable. Studies have shown that for patients with lymph node metastases, postoperative radiation therapy to the inguinal region and pelvis is beneficial in improving survival and reducing recurrence. Indications for radiation therapy include (1) patients with vulvar lesions that are too extensive to be surgically resected. Radiation therapy as preoperative treatment can reduce the extent of the lesion, decrease tumor cell activity, and increase the rate of surgical resection. (2) Patients who are too old and weak to tolerate surgery or have serious contraindications to surgery. (3) The surgical margin is not clean, or the surgical margin is too close to the tumor margin and postoperative radiotherapy. (4) Palliative radiotherapy for advanced and recurrent vulvar cancer can relieve symptoms and improve survival quality [1].

Due to the low incidence of vulvar cancer and the exact effect of initial surgical treatment, there are few clinical studies and a lack of evidence-based medical research on the application of chemotherapy alone for the treatment of vulvar cancer [17]. At present, clinically, chemotherapy is mostly used as adjuvant treatment to surgery or radiotherapy, for presurgical adjuvant treatment of locally progressive stages of vulvar cancer (such as stage III or IV) and for the combined application of chemotherapy and radiotherapy to patients who cannot be operated; or as postoperative adjuvant treatment, which can be used alone or combined with radiotherapy; or for treatment of recurrent vulvar cancer. Preoperative neoadjuvant chemotherapy is mainly used to control the primary tumor, reduce the size of the tumor, narrow the scope of surgical resection, or reduce surgery-related complications to facilitate subsequent treatment. At present, the commonly used chemotherapy regimens for vulvar cancer are mainly combination chemotherapy with cisplatin or 5-FU as the main drugs, including NF (HN2 + 5-FU) and PAB (DDP + ADM + BLM), which can be used in combination with radiotherapy and have good prospects for improving survival or life treatment of patients with moderately advanced or recurrent vulvar cancer. More clinical experience in chemotherapy of vulvar cancer still needs to be explored [18–20].

### 2.2. Laparoscopic Inguinal Lymph Node Dissection

Although laparoscopic inguinal lymph node dissection was first performed in vulvar cancer surgery, its safety and significant reduction of postoperative complications in the inguinal region were initially demonstrated by Mathevet et al. [21]. Since 2002, the subsequent use of laparoscopic inguinal lymph node dissection in vulvar cancer has rarely been reported. Some scholars have carried out laparoscopic inguinal lymph node dissection in patients with penile cancer and malignant melanoma of the lower extremities, drawing on the experience of laparoscopic techniques for lymph node dissection in breast cancer patients.

The low bleeding, low incidence of postoperative complications, and comparable number of lymph nodes resected with open surgery in laparoscopic surgery indicate that laparoscopic surgery is safe and feasible. Another index to evaluate the feasibility and safety of laparoscopic inguinal lymph node dissection is the postoperative tumor recurrence and 5-year survival of patients. Because laparoscopic inguinal lymph node dissection is an emerging technique, most of the current relevant studies are single-center studies with small sample sizes, and most of the articles are retrospective analyses without control groups and short follow-up times. Therefore, conducting prospective comparative studies with multicenter and larger samples will be under the direction of future research.

### 2.3. Nursing Method

Due to the special surgical site of vulvar cancer and the fact that the surgical incision is adjacent to the urethra and anus, it is very easy to be infected, easy to be moist locally, difficult to heal due to high tissue tension, and easy to form a cavity. The inguinal lymph node dissection under lumpectomy is less traumatic, has less bleeding, and is less painful, which avoids the problems of skin necrosis in the inguinal area, long-term poor healing of the incision, and the inability to carry out the subsequent treatment as scheduled and greatly shortens the hospital stay while reducing the damage. For the specificity of the surgical site, nursing care focuses on postoperative incision observation and care, guidance and feedback on patient activities, and appropriate psychological intervention, which are particularly important for patient recovery, and reasonable and effective treatment and care have important clinical significance [22, 23].

Psychological care: patients lack medical knowledge and are extremely concerned about the safety of surgery, incision pain, and prognosis. They are worried about the destruction of the vulva after surgery, which will seriously affect sexual life and the relationship between husband and wife. In order to reduce the patient's psychological burden, psychological care methods such as support and guidance are used to relieve the patient's psychological barriers, make him face reality correctly, and build up confidence.

Preoperative care: improve preoperative examination, exclude contraindications to surgery and anesthesia, and actively adjust blood pressure, blood sugar, and nutrition to improve the patient's tolerance to surgery. Keep the vulva clean and pay attention to prevent scratching the skin.

Intraoperative care: Keep the patient's thigh and abdomen on the same level, bend the knees, about 140° between the upper and lower legs, abduct the feet as much as possible to prevent the fibula capitulum from being in close contact with the leg support, the popliteal fossa is suspended, and the separation angle between the two legs is about 75°. This position is conducive to the exposure of the inguinal region and to keep the limbs in a functional position as much as possible when laparoscopic inguinal lymphatic dissection is performed. When wide vulvectomy is performed, the legs are adjusted to 100°∼120° apart, hip flexion 90°∼100°, and knee flexion 90°∼100°, which is conducive to exposing the vulva and facilitating the surgeon's operation; when closing the vulvar incision, the legs are adjusted to 70°∼80° apart to reduce the tension of the incision and facilitate the healing of the incision after surgery. Small soft pillows are placed on the buttocks and lumbar area. After inguinal lymph node dissection, send the lymph nodes for pathological examination in a timely manner and establish pneumoperitoneum for pelvic lymph node dissection if the result is positive [24].

Postoperative care: first-level care, diet ban, stay with a companion, rehydration, and oxygenation were given as prescribed by the doctor after surgery. Due to the richness of nerve endings in the perineum, the postoperative incision was wrapped with a large number of cotton pads with pressure, and the patient often felt pain and discomfort. To ensure the patient's comfortable postoperative activities and rest, an anesthetic analgesic pump was used as prescribed by the doctor, and the patient's attention was distracted by communicating with the patient and listening to soft music, and the nursing operation was concentrated as much as possible with gentle movements to allow the patient to rest fully at night. Complications in the inguinal lymphatic drainage area are mainly skin flap infection and necrosis, resulting in delayed healing of the incision. The incision should be taken care of to prevent bleeding. To prevent vaginal adhesions, iodoform gauze is placed in the vagina, and the vulvar incision is cleaned and disinfected with iodophor solution daily. After inguinal lymph node dissection on both sides, lymphatic fluid, tissue fluid, and exudate will inevitably accumulate under the skin flap, so the drainage tube should be taken care of in a timely manner. When caring for the urinary catheter, it should be kept open. Take care of their bowel movements.

Functional exercise and rehabilitation guidance: patients are prone to vaginal opening stenosis caused by incision scar or contracture due to surgical removal of large amount of tissues. After 7∼10 days postoperatively, functional exercises should be performed twice a day for 10∼20 minutes each time, such as closing, separating, forward flexion, back extension, abduction, and adduction of the legs, with gentle and slow movements and a range of activities from small to large. According to the patient's age and condition, the patient should be instructed to perform pelvic floor muscle contraction training to reduce scar contracture and improve urinary and bowel function.

## 3. Discussion

Vulvar cancer is a malignant tumor that occurs mostly in women. The clinical cause of this disease is not clear but is thought to be mainly related to genetic predisposition, excessive alcohol consumption, and the use of exogenous estrogens. In recent years, the incidence of this disease has been on the rise. Vulvar cancer itself does not affect patients' life and health, but it can adversely affect vital organs and structures such as the liver, lungs, and bone due to cell shedding and metastasis, which can lead to various symptoms and threaten patients' life and health. Surgery is the main treatment method for vulvar cancer patients. In the past, modified radical surgery was usually used in clinical practice, which is effective in removing cancerous tissues, but it is more traumatic and has a slower recovery rate, which has a greater impact on patients' psychology and quality of life [25, 26].

With the further improvement of laparoscopic instruments and technical development, laparoscopy has been widely used in the treatment of gynecological malignancies. Care of vulvar cancer surgery is also an important part of the success of surgery. We should strengthen patient psychological care before surgery, fully improve preoperative examination and assessment preparation, closely observe the condition after surgery, and conduct a good job of observation and prevention of postoperative complications. Because of the large amount of subcutaneous tissue removed during open resection of inguinal lymph nodes, long-term poor healing of the inguinal incision is likely to occur after surgery, with an incidence of more than 50% reported in the literature. Laparoscopic inguinal lymphatic dissection can effectively avoid the common problems of skin necrosis and long-term poor healing of the inguinal incision after open surgery because the surgery is performed in the subcutaneous space, and there is no incision in the skin of the inguinal region, which is less traumatic, the postoperative recovery is fast, and the hospital stay is shortened [5, 27].

## 4. Conclusion

In conclusion, the combination of radical vulvar cancer surgery with laparoscopic inguinal lymph node dissection with quality nursing intervention can promote patients' recovery, shorten the operation time, and reduce the incidence of patients' complications, which has significant clinical significance.

## Figures and Tables

**Figure 1:** Nursing mechanism of vulvar cancer radical surgery combined with laparoscopic inguinal lymph node dissection.

**Figure 2:** Read 121 articles, including 45 RCTs and 11 recommendations. Only 13 RCTs and 8 recommendations remained.

**Table 1:** Guidelines with high-level evidence and their impact size.

Organization	Guidelines with high standard of proof and effect size	
OARSI 2014 [22]	Exercise	Pain and function
	Weight loss	Pain and function
	Education	Pain

ESCEO 2014 [15]	Information/education	Treatment adherence
	Weight loss if overweight, exercise (strength training, aerobic training)	Function and pain
		Function and pain

NICE 2014 [18]	Education	Pain, function, and stiffness
	Exercise	Pain, function, and stiffness
	Weight loss	Pain, function, and stiffness
	Biomechanical interventions	Pain, function, and stiffness

AAOS 2013 [20]	Education	Pain
	Exercise	Function
	Weight loss	Disability
	Biomechanical interventions	Other symptoms

EULAR 2013 [14]	Education	Pain
	Exercise	Pain and function
	Weight loss	Pain and function
	Lifestyle changes	Pain and function

ACR 2012 [21]	Exercise	Pain and function
	Weight loss	Pain and function

RACGP NHMRC 2009 [19]	Weight loss	Pain and disability
	Exercise	Pain and function
	Education	Treatment adherence
		Pain and quality of life

SOFMER SFR SOFCOT 2008 [13]	Exercise	Pain and function
	Patient education and psychological support	Treatment adherence

## Data Availability

The experimental data used to support the findings of this study are available from the corresponding author upon request.
